# Effect of Acute Limb Ischemia on the Mortality of Patients with Extracorporeal Membrane Oxygenation Established by Femoral Vein-Arterial Catheterization and Analysis of Related Risk Factors

This article has been retracted.

**DOI:** 10.1155/2021/3471764

**Published:** 2021-08-30

**Authors:** Xiang Li, Guang Chen, Sheng Zhang, Xinting Zheng, Wenjun Zhao, Dun Hong

**Affiliations:** ^1^Department of Vascular Surgery, Taizhou Hospital Affiliated to Wenzhou Medical University (Zhejiang Province Taizhou Hospital), Taizhou 317000, Zhejiang, China; ^2^Department of ICU, Taizhou Hospital Affiliated to Wenzhou Medical University (Zhejiang Province Taizhou Hospital), Taizhou 317000, Zhejiang, China; ^3^Department of General Practice, Taizhou Hospital Affiliated to Wenzhou Medical University (Zhejiang Province Taizhou Hospital), Taizhou 317000, Zhejiang, China; ^4^Department of Orthopaedics, Taizhou Hospital Affiliated to Wenzhou Medical University (Zhejiang Province Taizhou Hospital), Taizhou 317000, Zhejiang, China

## Abstract

Extracorporeal membrane oxygenation (ECMO) is a common treatment for cardiopulmonary failure. Although it can effectively reduce the mortality of patients with cardiopulmonary failure, it still has a high mortality rate, such as acute limb ischemia (ALI), stroke, liver and kidney failure, and other related complications and related causes of death. This study aims to explore the impact of ALI on the mortality of VA-ECMO patients in hospital and 6 months after discharge and analyze the occurrence of ALI and related factors that affect the mortality of VA-ECMO in hospital and 6 months after discharge. The results showed that the smoking history was an independent risk factor for ALI, and age, diabetes, cardiac arrest, first time of ECMO, and hyperbilirubinemia were associated risk factors for in-hospital mortality. Cardiac arrest and ALI were associated risk factors for mortality at 6 months after discharge. Although ALI is not significantly associated with VA-ECMO in-hospital mortality, it is a risk factor for mortality at 6 months after discharge, and medical personnel should therefore strive to reduce and avoid ALI.

## 1. Introduction

Extracorporeal membrane oxygenation (ECMO) is a continuous extracorporeal vital sign treatment method, which uses extracorporeal equipment to replace or partially replace the human heart and lung functions, and supports life to fight for the chance of heart and lung disease healing and functional recovery [1, 2]. The two main configurations of ECMO currently in use are vein-venous (V-V) ECMO for respiratory support and vein-arterial (V-A) ECMO for cardiopulmonary support. For patients with cardiopulmonary insufficiency, V-A ECMO is the first choice of supportive treatment, which can provide comprehensive cardiopulmonary support. ECMO as a treatment for cardiopulmonary failure has grown exponentially over the past decade, and several landmark studies have shown that ECMO is effective in reducing mortality in cardiopulmonary failure [3, 4]. However, ECMO itself is not without major complications, and it still has a high mortality rate, such as acute limb ischemia (ALI), stroke, and liver and kidney failure, which are related complications and causes of death [5–8]. ALI is a common emergency in vascular surgery. If it is not treated in time, it can cause irreversible necrosis of the limbs and amputation and even endanger the life of the patient [9]. Therefore, it is extremely important to explore the risk factors of ALI in patients and prevent them. Although the ECMO patients survival has improved significantly, what factors affect mortality is still not clear, and there is still lack of relevant data and research on the impact of vascular complications on the prognosis of VA-ECMO patients, especially in the ischemic vascular complications of hospital mortality and six months after hospital discharge, mortality, and the influence of other complications [10–12]. This study aims to explore the impact of ALI on the mortality of VA-ECMO patients in hospital and 6 months after discharge and analyze the occurrence of ALI and related factors that affect the mortality of VA-ECMO in hospital and 6 months after discharge. The specific report is as follows.

## 2. Materials and Methods

### 2.1. Patients

A retrospective analysis of the clinical data of 124 VA-ECMO patients admitted to the ICU in our hospital from August 2017 to August 2020. Inclusion criteria: all received VA-ECMO treatment; survived more than two hours after VA-ECMO was initiated (regardless of whether there is cardiogenic shock or respiratory failure); clinical data are complete. Exclusion criteria: there are contraindications for ECMO supportive treatment; those with congenital heart disease; those with unrepaired aortic dissection; those with severe valve insufficiency; those who fall off during follow-up. This study was approved by the ethics committee of our hospital, and informed consent was signed by the patients and their families.

### 2.2. ECMO Support the Treatment Intubation Method

The specific intubation method of ECMO is the same as previous research reports [13]. The appropriate type of cannula was selected according to the height and weight of the patients, and single lumen cannula was used for venous and arterial catheterization. The right femoral artery is preferred for femoral artery intubation, and the left femoral artery intubation is used if the right femoral artery is used for other treatments or if ultrasound suggests other obstacles to intubation.

### 2.3. Research Method

Ischemic vascular complications were defined as ALI [14] with changes in lower limb symptoms (decreased skin temperature and loss of arterial pulsation) and loss of peripheral Doppler flow signals (vascular anastomotic repair during ECMO extubation was not included in the scope of vascular complications). Intervention options for ischemic vascular complications include open thrombolysis, intravascular interventional repair, fasciotomy decompression, or amputation. The ECMO team in our hospital is composed of doctors from ICU and vascular surgery. The femoral arteriovenous cannula is percutaneously punctured and cannulated by the vascular surgery assisting ICU doctor under the guidance of B-ultrasound. The process is managed by the ICU throughout the process, and the extubation is sutured by the ICU doctor assisting the vascular surgeon using the ProGlide suture device. If acute vascular complications occur during the period, the vascular surgeon is the mainstay, and the orthopedics and cardiothoracic surgery departments will assist in the rescue.

All patients were divided into the limb ischemia group and nonlimb ischemia group according to the presence or absence of ALI. The in-hospital mortality and the mortality 6 months after discharge were recorded and compared between the two groups. Age, sex, chronic medical history, ECMO intubation (catheterization method, type and location of the drainage tube and perfusion tube, and distal perfusion tube DPC), and other clinical data of all patients were recorded. The hospitalized death/survival status of the patients was recorded. The hospitalized surviving patients were followed up from the first day after discharge, and all were followed up for 6 months. The death/survival status was recorded through outpatient follow-up, telephone, or on-site follow-up.

### 2.4. Statistical Method

The results of this experiment were statistically analyzed by SPSS 20.0 (SPSS Co., Ltd., Chicago, USA). Normally distributed measurement data are represented by (mean ± standard deviation), and the *t*-test was used for their comparison between groups. Nonnormally distributed measurement data are represented by the median (25th percentile, 75th percentile) (M (P25, P75)), and the Mann–Whitney *U* test is used for analysis. Count data were expressed by (rate), and the chi-square test was used for their comparison between groups. Multivariate analysis adopts the multiple logistic regression model. *P* < 0.05 indicates that the difference is statistically significant.

## 3. Results

### 3.1. Univariate Analysis of Influencing the Occurrence of ALI in Patients

A total of 124 patients were included in this study, including 16 patients with acute limb ischemia (7 patients with open thrombectomy, 1 patient with fasciotomy and decompression, and 8 patients with family members who chose conservative palliative care) and 108 patients without limb ischemia. Univariate analysis showed that the smoking history was associated with ALI (*P* < 0.05), as given in Table 1.

### 3.2. Multifactor Analysis of Influencing the Occurrence of ALI in Patients

Multivariate logistic analysis showed that age, proportion of female, BMI, hypertension, diabetes, cardiac arrest, drainage tube model, perfusion tube model, drainage-perfusion tube ipsilateral, distal perfusion tube DPC, first auxiliary time of ECMO, and hyperbilirubinemia had no significant correlation with the occurrence of ALI (*P* > 0.05). Smoking history was an independent factor of ALI (*P* < 0.05), as given in Tables 2 and 3.

### 3.3. Outcome of ECMO Patients with the Limb Ischemia Group and Nonlimb Ischemia Group

In the limb ischemia group, 6 patients died in hospital, 9 patients died within 6 months after discharge, the in-hospital mortality rate was 37.50% (6/16), and the mortality at 6 months after discharge was 56.25% (9/16). In the nonlimb ischemia group, 50 patients died in hospital, 25 patients died within 6 months after discharge, the in-hospital mortality rate was 46.30% (50/108), and the mortality at 6 months after discharge was 23.15% (25/108). The mortality at 6 months after discharge of the limb ischemia group was higher than that of the nonlimb ischemia group (*P* < 0.05), as shown in Figure 1.

### 3.4. Univariate Analysis of Influence on Death in ECMO Patients

Among the 124 ECMO patients, 56 died in hospital and 68 survived in hospital. According to the death/survival of the patients, they were divided into the hospitalized death group and hospitalized survival group for analysis. Univariate analysis showed that age, diabetes, cardiac arrest, ECMO first auxiliary time, and hyperbilirubinemia were related to hospital death of ECMO patients (*P* < 0.05), as given in Table 4.

### 3.5. Multivariate Analysis of Factors Affecting the Death of ECMO Patients in Hospital

Multivariate logistic analysis showed that age, diabetes, cardiac arrest, ECMO first assist time, and hyperbilirubinemia were independent influencing factors of hospital death in ECMO patients (*P* < 0.05), as given in Tables 5 and 6.

### 3.6. Univariate Analysis of Mortality of ECMO Patients 6 Months after Discharge

Among 68 ECMO patients, 35 died and 33 survived 6 months after discharge. According to the death/survival of patients, they were divided into 6-month discharged death group and 6-month discharged survival group for analysis. Univariate analysis showed that cardiac arrest and ALI were related to death of ECMO patients at 6 months after discharge (*P*), as given in Table 7.

### 3.7. Multifactor Analysis of Mortality of ECMO Patients 6 Months after Discharge

Multivariate logistic analysis showed that cardiac arrest and ALI were independent factors influencing the death of ECMO patients at 6 months after discharge (*P* < 0.05), as given in Tables 8 and 9.

## 4. Discussion

In the past few years, the use of ECMO is more and more wide, and the use of ECMO in our hospital is also increasing year by year. However, ECMO is not without risks. Many factors are affecting the prognosis of patients with ECMO. The most important preoperative influencing factor for the prognosis of patients is the patient's basic condition, which is often not obvious at the beginning of ECMO. Once ECMO is officially initiated, complications often determine the prognosis of patients with ECMO [15, 16]. Vascular and neurological complications are probably the most devastating because of their irreversible nature and their clear association with mortality [17–20]. At present, there are various reports on the incidence of VA-ECMO vascular complications in the literature. The association between vascular complications and mortality has not been fully established, some studies have not established the association between ALI and mortality, and there is a wide range of opinions about what factors affect mortality in ECMO patients. There is also a wide variety of literature with conflicting conclusions and no guideline conclusion or expert consensus [21–24].

There is literature that age, history of diabetes, history of stroke, and history of peripheral arterial disease are predisposing factors related to limb ischemia in ECMO patients [25]. However, in this study, the predisposing factor related to limb ischemia was smoking history, and other related factors such as demographic characteristics, chronic disease history, and other complications were not significantly related to acute limb ischemia. Some literature believes that the lack of the distal perfusion tube (DPC) is a very important risk factor related to limb ischemia. A meta-analysis of 22 retrospective studies evaluating the impact of DPC on the risk of limb ischemia showed that although there was no statistically significant difference in mortality between the DPC and non-DPC cohorts, the DPC group reduced the incidence of absolute limb ischemia by 15.7% compared with the non-DPC group (9.74% vs. 25.42%) [26]. This study also wanted to verify the correlation between ECMO intubation and acute limb ischemia and mortality, which could be analyzed statistically from the existing data in our hospital. The results showed that there was no significant correlation between ECMO catheterization (precatheterization, percutaneous puncture, incision, and incision + puncture), size and length of the drainage tube and perfusion tube, placement position of two tubes, and DPC with ALI and mortality. There is a literature showing a higher mortality rate in patients with limb ischemia and a strong association between vascular complications and hospital mortality. In that literature cohort, the survival rate at discharge was 18% and 49% for patients with and without vascular complications by the multivariate analysis, with a hazard ratio of 2.17 (*P*=0.02) [27]. However, the results of this study showed that limb ischemia had no direct effect on in-hospital mortality, but was significantly associated with mortality at 6 months after discharge.

In this study, why is ALI a predictor of mortality at 6 months after discharge, but not of in-hospital death? In 16 patients with ALI, 8 of them were treated with open thrombectomy and fasciotomy and decompression, all of them survived and were discharged, 7 died 6 months after discharge, and 1 survived. 8 patients were treated conservatively, 6 died during hospitalization, and 2 died 6 months after discharge. Presumably, ALI was actually associated with in-hospital mortality, but the intervention of the vascular surgeon improved ALI and saved the patient's life, so the effect on in-hospital mortality was statistically reduced. It can be concluded that ALI has an impact on in-hospital mortality, but further data and evidence are needed to support this. Although specific perspectives and conclusions vary from literature to literature, there is a common view that ischemic vascular complications have a significant impact on mortality and prognosis in ECMO patients, so we believe that prevention is critical. Early diagnosis of ECMO patients at risk of acute limb ischemia through clinical examination, Doppler ultrasound, ECG monitoring, and angiography, thus enabling patients to achieve better outcomes and has received increasing attention [28]. Once limb ischemia is detected, immediate action should be taken to reverse ischemic vascular complications.

This study also has multiple limitations. (1) This is a single institution study and a retrospective study with a small sample size. (2) Considering the urgency of ECMO patients, peripheral artery-related diseases are often less considered in rescue, and the analysis of causes of vascular complications may be biased. (3) The placement of the ECMO tube and distal perfusion tube (DPC) is not standardized, but determined by the rescue physician.

## 5. Conclusion

Smoking history was an independent risk factor for ALI, while age, diabetes, cardiac arrest, first time of ECMO, and hyperbilirubinemia were associated risk factors for in-hospital mortality. Cardiac arrest and ALI were associated risk factors for mortality at 6 months after discharge. Although ALI is not significantly associated with VA-ECMO in-hospital mortality, it is a risk factor for mortality at 6 months after discharge, and medical personnel should therefore strive to reduce and avoid ALI.

## Figures and Tables

**Figure 1:** Outcome of ECMO patients with the limb ischemia group and nonlimb ischemia group. Note: compared with the limb ischemia group, *P* < 0.05.

**Table 1:** Univariate analysis of influencing the occurrence of ALI in patients.

Variables	*n*	The limb ischemia group (*n* = 16)	The nonlimb ischemia group (*n* = 108)	*P*
Age (year)	124	54.31 ± 11.75	58.63 ± 13.91	0.236
Proportion of female (%)	37	4 (25.00%)	33 (30.56%)	0.651
BMI (kg/m^2^)	124	24.32 ± 2.95	23.40 ± 2.54	0.194
Hypertension (%)	49	5 (31.25)	44 (40.74)	0.469
Diabetes (%)	25	2 (12.50)	23 (21.30)	0.413
Hyperlipidemia (%)	5	2 (12.50)	3 (2.78)	0.065
Long history of oral anticoagulants (%)	10	0 (0.00)	10 (9.26)	0.204
History of myocardial infarction (%)	9	0 (0.00)	9 (8.33)	0.231
Smoking history (%)	32	9 (56.25)	23 (21.30)	0.003
History of COPD (%)	1	0 (0.00)	1 (0.93)	0.699
History of chronic kidney disease (%)	2	0 (0.00)	2 (1.85)	0.583
Cardiac arrest (%)	81	12 (75.00)	69 (63.89)	0.383
ECMO catheterization method				0.479
Prepositioned (%)	6	0 (0.00)	6 (5.56)	
Percutaneous puncture (%)	105	13 (81.25)	92 (85.19)	
Incision (%)	3	1 (6.25)	2 (1.85)	
Puncture + incision (%)	10	2 (12.50)	8 (7.41)	
Drainage tube model (F)	124	22.00 (16.00, 18.00)	21.00 (15.00, 24.00)	0.089
Perfusion tube model (F)	124	16.00 (16.00, 18.00)	16.00 (15.00, 23.00)	0.245
Drainage-perfusion tube ipsilateral (%)	64	7 (43.75)	57 (52.78)	0.501
Distal perfusion tube DPC (%)	43	6 (37.50)	37 (34.26)	0.799
ECMO first auxiliary time (h)	124	115.00 (52.40, 192.30)	78.10 (0.50, 405.90)	0.085
Live out of the hospital (%)	68	10 (62.50)	58 (53.70)	0.509
Acute stroke (%)	6	0 (0.00)	6 (5.56)	0.334
Hyperbilirubinemia (%)	63	10 (62.50)	53 (49.07)	0.316

**Table 2:** Assignment for multivariate analysis of factors.

Factors	Variable	Assignment
Age	*X*1	Continuous variable
Proportion of female	*X*2	No = 0, Yes = 1
BMI	*X*3	Continuous variable
Hypertension	*X*4	No = 0, Yes = 1
Diabetes	*X*5	No = 0, Yes = 1
Smoking history	*X*6	No = 0, Yes = 1
Cardiac arrest	*X*7	No = 0, Yes = 1
Drainage tube model	*X*8	Continuous variable
Perfusion tube model	*X*9	Continuous variable
Drainage-perfusion tube ipsilateral	*X*10	No = 0, Yes = 1
Distal perfusion tube DPC	*X*11	No = 0, Yes = 1
ECMO first auxiliary time	*X*12	Continuous variable
Hyperbilirubinemia	*X*13	No = 0, Yes = 1

**Table 3:** Multifactor analysis of influencing the occurrence of ALI in patients.

Variables	*B*	S.E	Wald	*P*	OR	95% CI
Age	−0.023	0.058	1.843	0.235	0.977	0.941–1.015
Proportion of female	−0.277	0.304	0.498	0.651	0.758	0.227–2.524
BMI	0.124	0.105	2.216	0.196	1.132	0.938–1.365
Hypertension	0.414	0.231	0.815	0.471	1.513	0.491–4.657
Diabetes	0.639	0.547	0.608	0.421	1.894	0.401–8.938
Smoking history	1.559	0.682	7.538	0.005	4.752	1.598–12.131
Cardiac arrest	0.528	0.369	1.249	0.388	1.696	0.512–5.617
Drainage tube model	0.358	0.593	3.416	0.091	1.431	0.946–2.162
Perfusion tube model	0.248	0.169	1.725	0.263	1.281	0.830–1.975
Drainage-perfusion tube ipsilateral	−0.362	0.241	0.649	0.502	0.696	0.242–2.004
Distal perfusion tube DPC	−0.141	0.382	0.205	0.799	0.869	0.293–2.576
ECMO first auxiliary time	0.005	0.016	3.412	0.092	1.005	0.999–1.011
Hyperbilirubinemia	0.549	0.398	1.419	0.322	1.731	0.587–5.094

**Table 4:** Univariate analysis of influence on death in ECMO patients.

Variables	*n*	The hospitalized death group (*n* = 56)	The hospitalized survival group (*n* = 68)	*P*
Age (year)	124	61.91 ± 16.80	55.14 ± 9.45	0.006
Proportion of female (%)	37	18 (32.14)	19 (27.94)	0.611
BMI (kg/m^2^)	124	23.61 ± 2.15	23.42 ± 2.93	0.621
Hypertension (%)	49	22 (39.29)	27 (39.71)	0.962
Diabetes (%)	25	5 (8.93)	20 (29.41)	0.005
Hyperlipidemia (%)	5	1 (1.79)	4 (5.88)	0.248
Long history of oral anticoagulants (%)	10	3 (5.35)	7 (10.29)	0.315
History of myocardial infarction (%)	9	6 (10.71)	3 (4.41)	0.178
Smoking history (%)	32	11 (19.64)	21 (30.88)	0.155
History of COPD (%)	1	0 (0.00)	1 (1.47)	0.362
History of chronic kidney disease (%)	2	0 (0.00)	2 (2.94)	0.196
Cardiac arrest (%)	81	44 (78.57)	37 (54.41)	0.005
Drainage tube model (F)	124	21.00 (18.00, 24.00)	20.00 (15.00, 24.00)	0.322
Perfusion tube model (F)	124	16.00 (14.00, 17.00)	16.00 (15.00, 23.00)	0.075
Drainage-perfusion tube ipsilateral (%)	64	32 (57.14)	32 (47.06)	0.263
Distal perfusion tube DPC (%)	43	18 (32.14)	25 (36.76)	0.591
ECMO first auxiliary time (h)	124	37.50 (0.33, 296.20)	106.80 (10.30, 405.90)	0.001
Bleeding complications (%)	13	5 (8.93)	8 (11.76)	0.608
Acute stroke (%)	6	2 (3.57)	4 (5.88)	0.551
Hyperbilirubinemia (%)	63	36 (64.29)	27 (39.71)	0.006
ALI (%)	16	6 (10.71)	10 (14.71)	0.509

**Table 5:** Assignment for the multivariate analysis of factors.

Factors	Variable	Assignment
Age	*X*1	Continuous variable
Proportion of female	*X*2	No = 0, Yes = 1
BMI	*X*3	Continuous variable
Hypertension	*X*4	No = 0, Yes = 1
Diabetes	*X*5	No = 0, Yes = 1
Long history of oral anticoagulants	*X*6	No = 0, Yes = 1
History of myocardial infarction	*X*7	No = 0, Yes = 1
Smoking history	*X*8	No = 0,Yes = 1
Cardiac arrest	*X*9	No = 0, Yes = 1
Drainage tube model	*X*10	Continuous variable
Perfusion tube model	*X*11	Continuous variable
Drainage-perfusion tube ipsilateral	*X*12	No = 0, Yes = 1
Distal perfusion tube DPC	*X*13	No = 0, Yes = 1
ECMO first auxiliary time	*X*14	Continuous variable
Acute stroke	*X*15	No = 0, Yes = 1
Hyperbilirubinemia	*X*16	No = 0, Yes = 1
ALI	*X*17	No = 0, Yes = 1

**Table 6:** Multivariate analysis of factors affecting the death of ECMO patients in hospital.

Variables	*B*	S.E	Wald	*P*	OR	95% CI
Age	0.041	0.014	6.895	0.008	1.041	1.011–1.071
Proportion of female	−0.199	0.468	0.491	0.611	0.819	0.378–1.770
BMI	0.034	0.106	0.504	0.618	1.035	0.904–1.185
Hypertension	0.018	0.405	0.108	0.962	1.018	0.494–2.098
Diabetes	1.447	1.263	6.941	0.007	4.251	1.478–12.221
Long history of oral anticoagulants	0.707	0.954	0.765	0.323	2.027	0.499–8.235
History of myocardial infarction	0.956	0.988	1.059	0.192	2.601	0.620–10.909
Smoking history	0.603	0.406	1.518	0.157	1.828	0.792–4.218
Cardiac arrest	1.122	0.896	7.015	0.006	3.072	1.385–6.816
Drainage tube model	0.098	0.069	0.681	0.426	1.103	0.866–1.405
Perfusion tube model	−0.399	0.145	3.026	0.096	0.671	0.420–1.073
Drainage-perfusion tube ipsilateral	−0.405	0.106	0.912	0.264	0.667	0.321–1.359
Distal perfusion tube DPC	−0.205	0.219	0.524	0.591	0.815	0.368–1.719
ECMO first auxiliary time	−0.009	0.003	7.369	0.001	0.991	0.985–0.997
Acute stroke	0.523	1.168	0.583	0.555	1.687	0.298–9.572
Hyperbilirubinemia	1.005	0.751	6.952	0.007	2.733	1.316–5.679
ALI	0.363	0.615	0.602	0.511	1.437	0.488–4.233

**Table 7:** Univariate analysis of mortality of ECMO patients 6 months after discharge.

Variables	*n*	The 6-month discharge death group (*n* = 35)	The 6-month discharge survival group (*n* = 33)	*P*
Age (year)	68	56.10 ± 8.29	53.71 ± 9.08	0.262
Proportion of female (%)	19	8 (22.86)	11 (33.33)	0.336
BMI (kg/m^2^)	68	23.21 ± 3.06	23.59 ± 2.78	0.498
Hypertension (%)	27	14 (40.00)	13 (39.39)	0.959
Diabetes (%)	20	12 (34.29)	8 (24.24)	0.364
Hyperlipidemia (%)	4	3 (8.57)	1 (3.03)	0.332
Long history of oral anticoagulants (%)	7	2 (5.71)	5 (15.15)	0.201
History of myocardial infarction (%)	3	1 (2.86)	2 (6.06)	0.521
Smoking history (%)	21	13 (37.14)	8 (24.24)	0.249
History of COPD (%)	1	0 (0.00)	1 (3.03)	0.299
History of chronic kidney disease (%)	2	1 (2.86)	1 (3.03)	0.966
Cardiac arrest (%)	37	29 (82.86)	8 (24.24)	0.001
Drainage tube model (F)	68	20.00 (15.00, 24.00)	22.00 (18.00,24.00)	0.231
Perfusion tube model (F)	68	16.00 (15.00, 23.00)	16.00 (15.00,18.00)	0.495
Drainage-perfusion tube ipsilateral (%)	32	16 (45.71)	16 (48.48)	0.819
Distal perfusion tube DPC (%)	25	10 (28.57)	15 (45.45)	0.149
ECMO first auxiliary time (h)	68	106.80 (10.30, 218.60)	106.30 (43.75, 405.90)	0.129
Bleeding complications (%)	8	4 (11.43)	4 (12.12)	0.929
Acute stroke (%)	4	1 (2.86)	3 (9.09)	0.275
Hyperbilirubinemia (%)	27	15 (42.86)	12 (36.36)	0.584
ALI (%)	10	9 (25.71)	1 (3.03)	0.008

**Table 8:** Assignment for multivariate analysis of factors.

Factors	Variable	Assignment
Age	*X*1	Continuous variable
Proportion of female	*X*2	No = 0, Yes = 1
BMI	*X*3	Continuous variable
Hypertension	*X*4	No = 0, Yes = 1
Diabetes	*X*5	No = 0, Yes = 1
Long history of oral anticoagulants	*X*6	No = 0, Yes = 1
History of myocardial infarction	*X*7	No = 0, Yes = 1
Smoking history	*X*8	No = 0, Yes = 1
Cardiac arrest	*X*9	No = 0, Yes = 1
Drainage tube model	*X*10	Continuous variable
Perfusion tube model	*X*11	Continuous variable
Drainage-perfusion tube ipsilateral	*X*12	No = 0, Yes = 1
Distal perfusion tube DPC	*X*13	No = 0, Yes = 1
ECMO first auxiliary time	*X*14	Continuous variable
Acute stroke	*X*15	No = 0, Yes = 1
Hyperbilirubinemia	*X*16	No = 0, Yes = 1
ALI	*X*17	No = 0, Yes = 1

**Table 9:** Multifactor analysis of mortality of ECMO patients 6 months after discharge.

Variables	*B*	S.E	Wald	*P*	OR	95% CI
Age	0.031	0.056	0.962	0.259	1.032	0.977–1.091
Proportion of female	−0.523	0.359	0.815	0.338	0.593	0.203–1.729
BMI	−0.058	0.106	0.652	0.493	0.944	0.801–1.221
Hypertension	0.026	0.652	0.209	0.959	1.026	0.388–2.711
Diabetes	0.489	0.814	0.863	0.365	1.631	0.566–4.701
Long history of oral anticoagulants	1.081	0.903	0.817	0.339	2.946	0.530–16.379
History of myocardial infarction	0.786	1.165	0.592	0.531	2.194	0.189–25.402
Smoking history	0.614	0.912	0.966	0.253	1.847	0.646–5.281
Cardiac arrest	2.715	1.652	8.951	0.001	15.102	4.624–49.451
Drainage tube model	−0.185	0.138	0.946	0.232	0.831	0.613–1.126
Perfusion tube model	0.161	0.129	0.643	0.497	1.174	0.739–1.863
Drainage-perfusion tube ipsilateral	−0.111	0.264	0.329	0.819	0.895	0.345–2.321
Distal perfusion tube DPC	−0.732	0.258	1.469	0.152	0.481	0.176–1.311
ECMO first auxiliary time	−0.005	0.006	1.354	0.138	0.995	0.988–1.002
Acute stroke	1.224	1.581	0.886	0.302	3.401	0.336–34.453
Hyperbilirubinemia	0.272	0.846	0.532	0.585	1.312	0.495–3.481
ALI	2.405	1.952	5.126	0.027	11.077	1.317–93.192

## Data Availability

The data used to support the findings of this study are available from the corresponding author upon request.
